# Thermal Disproportionation for the Synthesis of Silicon Nanocrystals and Their Photoluminescent Properties

**DOI:** 10.3389/fchem.2021.721454

**Published:** 2021-08-12

**Authors:** Yize Su, Chenhao Wang, Zijian Hong, Wei Sun

**Affiliations:** ^1^ State Key Laboratory of Silicon Materials, School of Materials Science and Engineering, Zhejiang University, Hangzhou, China; ^2^ Lab of Dielectric Materials, School of Materials Science and Engineering, Zhejiang University, Hangzhou, China

**Keywords:** photoluminescence, silicon-rich oxide, thermal disproportionation, nanocrystals, quantum confinement, silicon

## Abstract

In the past decades, silicon nanocrystals have received vast attention and have been widely studied owing to not only their advantages including nontoxicity, high availability, and abundance but also their unique luminescent properties distinct from bulk silicon. Among the various synthetic methods of silicon nanocrystals, thermal disproportionation of silicon suboxides (often with H as another major composing element) bears the superiorities of unsophisticated equipment requirements, feasible processing conditions, and precise control of nanocrystals size and structure, which guarantee a bright industrial application prospect. In this paper, we summarize the recent progress of thermal disproportionation chemistry for the synthesis of silicon nanocrystals, with the focus on the effects of temperature, Si/O ratio, and the surface groups on the resulting silicon nanocrystals’ structure and their corresponding photoluminescent properties. Moreover, the paradigmatic application scenarios of the photoluminescent silicon nanocrystals synthesized via this method are showcased or envisioned.

## Introduction

It has been almost 30 years since the discovery of silicon nanocrystals (SiNCs) (Canham, 1990), which carry unique properties distinct from bulk silicon. Since then, SiNCs have gained enormous attention around the world and harvested countless achievements in a myriad of hot fields (Kubby et al., 2006; Liang and Bowers, 2010; Mastronardi et al., 2012a; Bonafos et al., 2012; McVey and Tilley, 2014; Zhai et al., 2014; Sun et al., 2016c; Dasog et al., 2016; Meinardi et al., 2017; Ni et al., 2019). Many of the applications are based on SiNCs’ photoluminescent properties. Consequently, significant progress has been achieved in the performance of their photoluminescence (PL) with the concerted efforts by the numerous nanochemists and physicists: the quantum yield (QY) has risen from a few percentages to more than 70% (Sefannaser et al., 2021), and the photoluminescence window has been expanded to a full range from ultraviolet to infrared (Hessel et al., 2012; Ghosh and Shirahata, 2014). Among the many factors that helped to find the PL benchmarks of SiNCs, the preparation or synthetic method plays a primary and pivotal role.

Similar to many other widely used nanomaterials, SiNCs can be prepared with versatile methods, and each of them has its own advantages and challenges. For example, electrochemical etching, one of the earliest methods for preparing SiNCs (Cullis and Canham, 1991), sacrifices the controllability of size to realize simplicity (Heinrich et al., 1992; Bley et al., 1996). Similarly, laser ablation also faces the challenge of controllability, and the requirement of sophisticated equipment hinders its adoption by chemical labs, but its facile route allows fabrication in one step with little waste (Shirahata et al., 2009b; Mangolini, 2013; Krivonosov et al., 2020). Another synthetic method demanding for specialized equipment is plasma synthesis, of which the high yield and surface hydride termination have drawn considerable interest (Mangolini et al., 2005; Liu et al., 2016; Chen et al., 2020b). Besides, solution-phase synthesis has the advantages of high productivity and feasibility (Shirahata et al., 2009a; He et al., 2011; Atkins et al., 2012; Ma et al., 2016). However, some researchers have raised the concern that carbon impurities could have been incorporated into the product (Oliinyk et al., 2019; Ddungu et al., 2020; Wilbrink et al., 2020). In this context, if one is seeking the combined merits of tunability in size, relatively high production yields without carbon contamination, and concise processing procedures, then thermal disproportionation of silicon-rich oxides might be a suitable option. This eminent method has been widely utilized to enable the investigations of SiNCs’ chemical and physical properties.

The foundation of thermal disproportionation (in some reports referred to as “pyrolysis”) is rooted in the properties of silicon-rich oxide (some materials include H element as well) which would be decomposed to silicon and silicon dioxide under high-temperature treatment (above 900°C). The products’ figures of merits, especially photoluminescence properties, can be feasibly predetermined and adjusted during the thermal process. In addition, when freed from the oxide, the SiNCs prepared this way are often capped with active surface hydride groups, which enable further surface functionalization (Dasog et al., 2014; Chen et al., 2017).

Based on the advantages above, it is important to figure out the underlying contributor to the photoluminescent properties of SiNCs synthesized via the thermal disproportionation reaction. In this review, we first describe the basics of the thermal process and then discuss several key factors that dominate the properties of the resulting products, including size, temperature, composition, defects, and surface group. Finally, some paradigmatic applications of SiNCs synthesized via the thermal disproportionation reaction with appreciable photoluminescent properties are highlighted.

## Heating Process

The dynamic conversion process between the initial and final stage often remains a mystery, although it might be easier to identify the raw materials and final products of thermal disproportionation. Researchers have made great efforts to reveal the truth. The most studied precursor for the thermal disproportionation method is hydrogen silsesquioxane (HSQ), of which the pyrolysis was proposed to experience three stages (Figure 1A). When the temperature was lower than 400°C, HSQ began to cross-link, and the cage network was redistributed with associated loss of SiH_4_, but the definitive assignment of structural changes still required further research. Next, as the temperature rose from 500 to 900°C, amorphous Si nanodomains were formed and dehydrogenated. The source of Si nanodomains remained unclear, but it was possibly from SiH_4_. Only when the temperature was higher than 900°C, the crystalline products could be obtained. The pyrolysis process could also be further divided into five stages including trace solvent loss and collapse of pore structure unmentioned before (Hessel et al., 2006). The pictures of HSQ heated at different temperature were illustrated (Figure 1B). Besides, during rapid heating, the released SiH_4_ could not escape from the quickly formed SiO_2_ matrix before decomposition, which may enhance the productivity.

**FIGURE 1:** **(A)** Three stages of the thermal disproportionation process from room temperature to 1,400°C for HSQ, reprinted with permission from Hessel et al. (2007). Copyright 2007 American Chemical Society. **(B)** Photographs of HSQ heated at 500, 600, 700, 800, 900, 1,000, and 1,100°C for an hour respectively **(top** to **bottom)**, as prepared **(right)** and finely ground **(left)**, reprinted with permission from Hessel et al. (2006). Copyright 2006 American Chemical Society. **(C)** Schematic diagram of core-shell structured SiNCs with a model of the first ten atomic layers, reprinted with permission from Thiessen et al. (2019). Copyright 2019 American Chemical Society.

With the structure similar to HSQ which has the formula of HSiO_1.5_, the cross-linked (HSiO_1.5_)_*n*_ sol−gel polymer could undergo stages of Si cluster nucleation and crystallization, and above 1,100°C evident formation of SiNCs was observed (Henderson et al., 2009). Such polymer can be feasibly synthesized in a chemistry lab via the hydrolysis of common silane precursors (e.g., trichlorosilane); thus, the thermal disproportionation of it has been adopted as an economic alternative to the expensive commercial HSQ, for the synthesis of SiNCs with the diameter of several nm (Mastronardi et al., 2011; Mastronardi et al., 2012b; Sun et al., 2013).

However, the presence of Si-H bond seems not to be the prerequisite for the generation of SiNCs, as other silicon-rich oxide precursors can disproportionate. For instance, the conversion of microstructure within SiO from nanocluster to nanocrystal during pyrolysis was studied (Wang et al., 2007). When the temperature was below 300°C, a single random-bonded SiO-like phase was present; then, amorphous silicon-rich nanoclusters emerged and grew larger as the temperature rose from 400°C to 800 °C because of the exsolution of excess silicon. Finally, at a critical point between 800–900°C, silicon began to crystalize.

As for the heating process of silicon-rich oxide in the form of film, a theory of two thermal disproportionation stages was proposed, namely the precipitation of Si when the temperature was above 500°C and the crystallization of excess Si with the even higher temperature starting from ∼1,000°C (Gan et al., 2011). Since the PL had a close relationship with the size of SiNCs rather than that of amorphous silicon, the crystallization temperature therefore mattered (Thiessen et al., 2020). Amorphous materials cannot crystalize until the temperature reaches the threshold value. Below the threshold temperature, materials exist in the form of nanocluster, whose size increases with rising temperature. A diffusion kinetic model was built to explain the phenomenon which indicated that the diffusion coefficient has no relevance with composition (Nesbit, 1985), so the growth of size depends mainly on temperature.

Echoing with what we stated at the beginning of this section, it is quite obvious that the final products after very high-temperature treatment are the mixtures of SiNCs and SiO_2_, but what are the structure and composition of nanoclusters and their surrounding matrix before crystallization occurs? Here we discuss some more studies aiming at lower treating temperatures to help illustrate this aspect.

For example, heating siloxene, which can be seen to have the formula of Si_6_O_3_H_6_, at 400 °C for 90 min, could result in amorphous silicon dioxide embedded with small particles of amorphous silicon (Stutzmann et al., 1993). For precursors without H, Meldrum’s group revealed that the matrix for the Si clusters is not pure SiO_2_ if the reaction was incomplete, but is instead a mixture of SiO_2_ and SiO for the whole temperature range (Wang et al., 2007). In order to get a deeper understanding of the reaction process, the mechanism of transition from silicon-rich oxide to SiNCs was explored with the help of quantum mechanics and Monte Carlo (MC) simulation (Grimme et al., 2007). The result showed the driving force of pyrolysis conversion was mainly the incomplete O coordination, accompanied by strain as a minor contributor. O diffusion played a key role in controlling the reaction instead of excess Si diffusion.

All in all, we may not have covered all kinds of silicon-rich oxide precursors, but whether the precursor contains H or not, the thermal disproportionation generally follows the similar process. It can be compartmentalized into stages like the structural rearrangement, growth of the nanocluster or nanodomains, and finally crystallization of amorphous silicon which is often marked by a threshold temperature. Upon close examination, the SiNCs obtained are considered to possess the structure of crystalline core inside an amorphous shell (Figure 1C) (Borrero-Gonzalez et al., 2011; Thiessen et al., 2019).

## Factors on Photoluminescence

Needless to say that the photon of photoluminescence originates from the combination of electrons and holes. For direct bandgap materials like CdSe, the bottom of the conduction band fits the top of the valance band, resulting in efficient photoluminescence and nanosecond lifetime. However, limited by the indirect bandgap nature such that holes and electrons possess different k values (crystal momentum) in the Brillouin zone, bulk silicon can hardly emit light. However, decreasing its size to a few nanometers smaller than the Bohr radius (∼5 nm), silicon nanocrystals amazingly exhibit photoluminescence. The mechanism of this incredible phenomenon remains controversial. Many hypotheses have been put forward, such as the quantum confinement model (Canham, 1990), quantum confinement-luminescence center model (Qin and Jia, 1993; Qin and Li, 2003), and photoluminescence related to Si/SiO_2_ interface defects (Torchynska et al., 2003). Among them, the quantum confinement effect model is the most widely acknowledged hypothesis, despite the fact that other PL mechanisms are also proposed by researchers according to their concrete research. During the following sections, some of these mechanisms would be leveraged to elucidate the astonishing PL phenomena with details, but, experimentally, the PL performance of SiNCs predominantly depends on the major influencing factors categorized below, which should be comprehensively understood for the future development of SiNCs.

### Size

According to the quantum confinement effect, the band structure of nanoparticles is different from that of bulk materials. When the geometric radius of SiNCs reduces to lower than the radius of Bohr’s exciton, the energy levels of the valence band and the conduction band would change from continuous to discrete, and this broadens the energy bandgap. Accordingly, with the decrease of the SiNCs’ size, the absorption and fluorescence peaks blueshift (Sykora et al., 2008; Prokofiev et al., 2009; Kelly et al., 2010a; Kelly et al., 2010b). A number of groups have observed and revealed this relationship between PL energy or wavelength and the sizes of SiNCs (Figures 2A,B).

**FIGURE 2:** **(A)** PL peak energy versus diameter of SiNCs and the curve corresponds to the effective mass approximation (EMA), reprinted with permission from Hessel et al. (2012). Copyright 2012 American Chemical Society. **(B)** PL wavelength in visible range (solid line) and NIR range (dashed line) versus diameter of SiNCs and the inset shows the summary of PL center versus fraction number, reprinted with permission from Mastronardi et al. (2012). Copyright 2011 American Chemical Society. **(C)** Mechanism of the SiNCs photochemical etching by HF, reprinted with permission from Rodríguez Núñez et al., 2012. Copyright 2011 American Chemical Society. **(D)** AQY versus volume of antisolvent used and the corresponding size of SiNCs shown in the inset, reprinted with permission from Sun et al. (2015). Copyright 2014 WILEY-VCH Verlag GmbH & Co. KGaA, Weinheim.

In order to fabricate SiNCs with different size distributions, heating temperature and time are the first options that are effective and feasible. Generally both higher temperature and longer heating time would result in larger nanocrystals (Borrero-Gonzalez et al., 2011), but the temperature especially played a more crucial role among the two factors (Gan et al., 2011). For example, 3.3 nm of SiNCs was found after the disproportionation of HSQ at 1,100°C for 60 min. Raising the processing temperature to 1,400 °C could result in a relatively large size of 8.7 nm, but prolonging the processing time to 1,440 min at 1,100°C could only increase the size to 3.6 nm (Hessel et al., 2007). Alternatively, after the formation of SiNCs, a posttreatment of HF etching could also adjust SiNCs’ size distribution subsequently. The HF etching not only removes the concomitant oxides from the thermal disproportionation method, but also reduces SiNCs’ diameter. However, the etching reaction between Si and HF exhibited slow reaction kinetic process that hindered its application in reality. In this regard, the photochemistry etching method developed by Kolasinski (Kolasinski, 2003), Reipa (Choi et al., 2007), and Veinot (Rodríguez Núñez et al., 2012) et al. improved this situation and accelerated the etching process by treating the SiNCs in HF solution under the irradiation of light (Koyama and Koshida, 1993; Mizuno et al., 1996). Unlike the traditional chemistry etching that required an electronegative atom (e.g., O, F) bonding to Si to initiate the etching process, the photochemistry etching instead polarized the surface silicon by the localization of holes, which drove the nucleophilic attack (Figure 2C). As the photochemistry etching continuously progressed, the size of SiNCs could only be reduced to a limiting value and no further dissolution would occur afterwards (Choi et al., 2007). It was probably because the band gap of SiNCs increased as the size shrunk until the band gap was larger than the photon energy. In addition, the photochemistry etching process not only provided a novel method to adjust the PL, but also guaranteed the narrow size distribution with a full width at half maximum (FWHM) of PL peak as low as 90 nm, which is comparable to some of the lowest records reported (Rodríguez Núñez et al., 2012).

As for the relationship between the size and QY, taking the most-studied HSQ as an example, it was heated within the temperature range from 1,100 to 1,400 °C in a reducing atmosphere (10% H_2_ + 90% Ar) to obtain the SiNCs with a wide size distribution from under 3–90 nm, all of which were treated by similar surface passivation (Hessel et al., 2012). The photoluminescence test result revealed that the emission peak ranged from 720 nm for the size of 3 nm to 1,060 nm for the size of 12 nm, and the QY accordingly decreased from 8 to 0.4%, which is accorded with the quantum confinement model. Beyond the size of 12 nm, the bandgap of SiNCs closely approached that of the bulk silicon; thus, the PL of SiNCs could be hardly measured. Numerous researchers came to the similar conclusion which was coincident with the quantum confinement model, but some experiment results indicated the inverted trend of the PL QY versus size. Ozin’s group (Mastronardi et al., 2012b) found the AQY of small allylbenzene-capped SiNCs instead monotonically decreased as the size of SiNCs decreased from 2 to 1 nm, despite the fact that the PL peaks still blueshifted with the decreasing size, following the rules of quantum confinement. To explore the reason for this puzzling controversy, SiNCs were prepared with a series of size distributions from 2–7 nm with the help of size-selective precipitation, covering the whole size regime that possesses the strong quantum confinement effect (Sun et al., 2015). The result was surprising. As the size of SiNCs decreased monotonically, the AQY of these materials first increased and then fell after reaching the highest point, exhibiting a “volcano” plot (Figure 2D). The peak of the plot was obtained with SiNCs of 3 nm, in view of the fact that the luminescence lifetime (τ) and quantum yield (QY) are determined by the mutually competing radiative *Γ*_*r*_ and nonradiative *Γ*_*nr*_ rates of excitons, as illustrated in

$$\tau^{-1}=\Gamma_{r}+\Gamma_{nr}$$ (1)

$$QY=\Gamma_{r}/\left(\Gamma_{r}+\Gamma_{nr}\right)$$ (2)

PL lifetimes were measured to figure out the change of radiative relaxation. It turned out that PL lifetime decreased as the particle size decreased from 2 to 1 nm (Mastronardi et al., 2012b). The analysis combining the QY and lifetimes indicated the significant difference between the radiative recombination and nonradiative recombination. Specifically, the nonradiative recombination decreased dramatically more than radiative recombination as the size was smaller. Thus, the nonradiative recombination played a dominant role during the falling apart (left side) of the “volcano” plot in the low size regime. The attenuation of low-temperature lifetime compared with room-temperature lifetime further indicated that the drop of nonradiative recombination came from the vibration organic-capping group and oxidation-related defects. As for the right side of the “volcano” plot with larger size, when size decreased, the more confined spatial distribution of photogenerated electron-hole pairs was beneficial to radiation recombination and photon escapement; therefore, radiative recombination was instead dominant in this regime, resulting in the inversed trend compared to the left side of the volcano plot. The peak position of the “volcano” plot may change slightly for different materials, but the overall trend is in common (Riabinina et al., 2006; Yu et al., 2017).

### Composition

Silicon-rich oxide as the only reactant and precursor in the disproportionation reaction directly determines the proportion of the SiNCs in the products, so the composition of this precursor, particularly the Si/O ratio, has an enormous influence on the products. For instance, Sun found that the mass yield of SiO was more than twice that of (HSiO_1.5_)_n_ because of the higher Si/O ratio (Sun et al., 2016b). Meanwhile, the Si/O ratio can ultimately determine the threshold heating temperature for the synthesis of SiNCs (Dvurechensky et al., 1982). If silicon-rich oxides in the form of thin film are defined as SiO_x_, then when x < 1, it requires only 850 °C with a heating time of 1 h in the Ar atmosphere to obtain SiNCs, whereas when x is between 1 and 2, there is no appearance of SiNCs until the temperature hits the value of 1,050 °C. In another similar study, the minimum temperature of crystallization for Si/O ratio higher than one was between 800 and 950°C, but higher than 950°C for Si/O ratio less than 1 (Nesbit, 1985). In a word, at the same heating temperature, SiNCs obtained from a SiO_x_ precursor with a smaller x would be with larger size, better crystallization, and thereby redshift of PL peak position (Figure 3A) (Riabinina et al., 2006; Borrero-González et al., 2010; Saxena et al., 2011).

**FIGURE 3:** **(A)** Room-temperature PL spectra for annealed Si_y_O_1-y_ at 1,100°C in a forming atmosphere with different y, reprinted with permission from Borrero-González et al. (2010). Copyright 2010 American Institute of Physics. **(B)** Integrated PL intensity of P-doped SiNCs as a function of P concentration, reprinted with permission from Mimura et al. (2000). Copyright 2000 American Physical Society.

Note that even if the precursors are with the same Si/O ratio, their structural discrepancy can lead to variance in the product. HSQ and (HSiO_1.5_)_n_ have the same Si/O ratio, but are composed with different molecular structures. Under the same pyrolysis condition, it turned out that the SiNCs obtained from the former possessed a larger size than the latter (Henderson et al., 2009). The explanation was that the atom diffusion within the (HSiO_1.5_)_n_ cross-linked network required higher energy, which would hinder the formation and growth of SiNCs.

Another situation is when the precursor is not purely constituted by Si, O, and H. It is well known that doping with a small amount of group Ⅲ and Ⅴ elements such as B and P would dramatically influence the electrical properties of silicon wafer. As for the SiNCs with only a few nanometers in size, even a single impurity atom would make a difference in the optical and electrical properties of SiNCs. Boron and phosphorus are the most used dopants in the silicon-rich oxides and thereby in the product SiNCs. Their accompanied charge carriers after doping are opposite. However, their effects on PL are somehow similar: both boron-doped and phosphorus-doped SiNCs exhibited decreased PL intensities compared with pure SiNCs under the same excitation condition. The nonradiative Auger recombination induced by B or P doping was accounted for the drop of PL in the doped SiNCs (Mimura et al., 1999; Mimura et al., 2000; Joo et al., 2019). However, upon closer examination, the PL of P-doped SiNCs first increased to a maximum and then decreased as the P concentration further increased (Figure 3B). The temporary enhancement of P-doped SiNCs’ PL was because the stress at the interface between SiNCs and SiO_2_ matrix, which was induced during the cooling process after thermal disproportionation, was released by incorporating the P atoms into the matrix (Fujii et al., 1999). Although the doping of individual B or P into SiNCs would result in the quenching of PL, doping both B and P into SiNCs simultaneously could lead to the opposite result. The opposing charge carriers originated from the doping of B and P could be mutually compensated, which would avoid the Auger recombination. Therefore, the strong suppression of PL intensity would not occur in this case. Instead, enhanced PL intensity after codoping better than the pure SiNCs was observed, explained by two reasons. First, the softening of SiO_2_ matrix caused by the doping of B and P would reduce the stress of the products obtained after the annealing process and prevent the appearance of defects between the interface of SiNCs and SiO_2_. The other reason was that the electrons supplied by the P doping passivated the surface dangling bonds (Fujii et al., 2004). Those two mechanisms worked concertedly to enhance the PL intensity of B and P codoped SiNCs. In addition, the stability and dispersibility of the codoped SiNCs in polar solvents were also strengthened. The B and P codoped SiNCs maintained to be stable in methanol over one year and no precipitates were formed. A model was established to explain this phenomenon. The codoping of B and P formed P-B pairs within the SiNCs, and the B ions were located on the surface side whereas the P ions were on the core side. Therefore, the codoped SiNCs exhibited negative surface potential, which guaranteed the electrostatic repulsion for the high stability and dispersibility in methanol (Sugimoto et al., 2012). Besides, metal elements could also function as dopants (Wang et al., 2020; Xu et al., 2021a). Shirahata’s group synthesized metal- (Mn, Ni, Co, Cu) doped SiNCs accompanied by a redshift of PL while maintaining the relative high QY of 26% for codoping (Chandra et al., 2017). The metal elements within the SiNCs created new impurity states near the valence band, which resulted in the redshift of PL. Moreover, the narrower size distribution of transition-metal-doped SiNCs than the pure SiNCs was another advantage for this method.

### Defects

After thermal disproportionation of silicon-rich oxide, many defects emerged at the interface between SiNCs and SiO_2_, as the result of mismatch of the crystal structure and the dangling bonds. *P*_*b*_ center is a typical kind of defect that is widespread at these interfaces, which accounted for many nonradiative recombinations. *P*_*b*_ centers, the neutrally charged and paramagnetic dangling bonds, are the dominant charge traps at the interface between SiNCs and SiO_2_. Depending on its Fermi level in the silicon bandgap, it would either lose or gain an electron (Brower, 1988). As the nonradiative recombination centers, *P*_*b*_ defects would reduce PL intensity of SiNCs undoubtedly. Hence, it is necessary to passivate the *P*_*b*_ centers to obtain SiNCs with excellent PL.

In one study, SiNCs were prepared by annealing the Si implanted SiO_2_ at the temperature of 1,100°C in a N_2_ atmosphere for 1 h; then, the sample was passivated in the forming gas (95% N_2_ + 5% H_2_) at 500°C for another hour (Cheylan and Elliman, 2001). The resulting PL of SiNCs/SiO_2_ was effectively promoted after passivation. A redshift was also observed (Figure 4A) (Borrero-Gonzalez et al., 2011). Since larger SiNCs were likely to contain more defects, the positive influence of passivation was more effective for larger SiNCs than the smaller ones (Borrero-Gonzalez et al., 2011). Moreover, the passivation process was even reversible. Heating the passivated samples in the N_2_ atmosphere at ∼500°C could regenerate dangling bonds at the interface, which resulted in the decrease of PL intensity with blueshift. The PL performance could be completely reversible during the reciprocation of passivation and depassivation after the first three circles (Li et al., 2014b). Alternatively, the UV irradiation could also reintroduce defects for depassivation (Godefroo et al., 2008).

**FIGURE 4:** **(A)** PL spectra of SiNCs/SiO_2_ after annealing at 1,100 °C in N_2_ (□) and after an additional anneal at 500°C in forming gas (N_2_+H_2_) (○). The spectrum for the sample annealed at 1,100 °C in N_2_ has been multiplied by a factor of 5 to highlight the redshift (△). The solid lines represent the Gaussian fit to the data, reprinted with permission from Cheylan and Elliman. (2001). Copyright 2001 American Institute of Physics. **(B)** PL intensity of SiNCs/SiO_2_ at 1.7 eV **(left axis)** and the SiNCs’ mean size from TEM analysis **(right axis)** vs. annealing time at 1,100°C in N_2_, reprinted with permission from López et al. (2002). Copyright 2002 American Institute of Physics.

To study the influence of temperature and heating time of passivation, amorphous SiO_x_ was annealed at 1,100°C for 1 h and then postannealed in the forming gas at the varying temperature ranging from 400 to 700°C with the passivation time varying from 5 to 60 min (Li et al., 2014b). The result indicated that the higher the temperature, the greater the PL intensity, until the PL intensity saturated near 600°C and no further improvement of PL intensity was observed at 700°C. Similarly, the PL intensity first increased and gradually reached a constant value with the prolonging heating time. The saturation of the PL intensity at high temperature and long time could be explained by the balance of passivation and depassivation. The passivation mentioned above was achieved by the reaction between hydrogen molecules (H_2_) and dangling bonds. However, due to the steric hindrance of the interface structure between SiNCs and SiO_2_, the hydrogen molecule was too large to contact with exceptional dangling bonds. Therefore, using hydrogen atoms (single H) for passivation, whose volume was smaller than H_2_, could further improve the PL intensity. With this concept, postmetallization annealing (Wilkinson and Elliman, 2003) and H atomic plasma (Jung et al., 2008) were two effective methods to realize hydrogen atomic passivation. Nevertheless, the complicated process of atomic passivation limited its application, though it benefited the enhancement of PL intensity.

The passivation effect is also seen with annealing in oxygen atmosphere (Yoon, 2011). However, the situation changed for overtreatment. SiNCs embedded SiO_2_ samples were first annealed in N_2_ atmosphere at 1,100°C and then passivated in dry air flow at temperatures ranging from 400 to 800°C for 15–90 min (Li et al., 2014a). When the passivation temperature was below 600°C, the effect was roughly the same as hydrogen passivation: the PL intensity was first improved and then gradually saturated as the temperature and passivation time increased. However, the PL intensity started to fall when the temperature was above 600°C. In addition, at 800°C, the PL intensity first increased to a maximum for 0.5 h of passivation and next decreased accompanied by a blueshift as the time was prolonged. Such different phenomena can be attributed to the oxidation of SiNCs (Brongersma et al., 1998). The oxygen not only could passivate the dangling bonds, but also could oxide SiNCs, which resulted in the shrinkage of size and reduced number of SiNCs. At temperatures higher than 600°C, the oxidation effects instead of passivation played a dominant role, which resulted in the decrease of PL intensity.

Therefore, passivation is an excellent choice if the proper conditions are selected, to strengthen the PL for the merits of both the enhancement of PL intensity and the conservation of SiNCs’ structure (Figure 4B) (López et al., 2002; Li et al., 2014a). However, the passivation procedure complicates the production process. Hence, many researchers use a one-step compromising method that directly annealed the amorphous silicon-rich oxide in forming gas (e.g., 5% H_2_ in Ar or N_2_) to produce SiNCs embedded SiO_2_ with passivated interface, removing the extra passivation steps (Hessel et al., 2012; Yang et al., 2014; Thiessen et al., 2019).

### Surface Modification

Surface modification is a powerful technique to grant many nanomaterials with colloidal dispersibility and tunability of optical properties, and this is especially true for SiNCs.

The first merit of modification process is that it improves the PL stability. This is exemplified by ensembles covalently modified with alkynes and alkenes which are the most used ligands for functionalizing SiNCs through hydrosilylation. The prevention of oxidation and passivation of surface defects were the two main reasons that account for the improvement of stability after modification (Liu et al., 2006). The longer carbon chain length was particularly favorable in this regard for better oxidative and optical stability (Clark et al., 2010). Another way to produce SiNCs with superior stability was incorporating the SiNCs into surfactants, e.g., a structure where SiNCs were covered with a monolayer of quatsomes (Silbaugh et al., 2017) (Figure 5A). The quatsomes were vesicular bilayers self-assembled by cholesterol and cetyltrimethylammonium bromide (CTAB) surfactants. The products obtained by the combination of SiNCs and quatsomes could remain stable after several weeks in water with the conservation of PL of SiNCs.

**FIGURE 5:** **(A)** Scheme of the interactions of SiNCs (solid points) and quatsomes (CTAB is the blue-headed structure, and cholesterol is the yellow structure), and the formation of the stable SiNCs covered with a monolayer of quatsomes, reprinted with permission from Silbaugh et al. (2017). Copyright 2017 American Chemical Society. **(B)** PL spectral of SiNCs with different size and functionalized with NH_4_Br and allylamine, reprinted with permission from Wolf et al. (2013). Copyright 2013 American Chemical Society. **(C)** Schematic representation of the synthesis process of pyrene-functionalized SiNCs, reprinted with permission from Mazzaro et al. (2015). Copyright 2015 American Chemical Society. **(D)** The pictures of SiNCs/PMAA under the irradiation of ambient light **(top)** and UV **(bottom)**. From **left** to **right** were pure PMAA, H-terminated SiNCs/PMAA with smaller SiNCs and bigger SiNCs, and dodecene-terminated SiNCs/PMAA with smaller SiNCs and bigger SiNCs, reprinted with permission from Marinins et al. (2016). Copyright 2016 American Chemical Society.

Second, surface modification can shift the PL position. In retrospect, we emphasized that the size matters for the peak position, but the ultimate surface functionalization can disrupt or even override the size effect. As an example, different capping groups including alkynes, phenylacetylene, 4-ethynylanisole, 1-ethynyl-3-fluorobenzene, and 3-ethynylthiophene were functionalized with SiNCs (Kelly and Veinot, 2010), and their PL behaviors were investigated. The PL decay rates of the functionalized SiNCs were contingent on the electron donating ability of organic ligands. The stronger the electron donating ability of substituents, the faster the decay rate of photoluminescence. Complete PL quenching was even observed for SiNCs functionalized with 3-ethynylthiophene. In another study, redshift was observed after modification with similar capping groups: after modifying SiNCs with phenylacetylene, 2-ethynylnaphthalene, and 2-ethynyl-5-hexylthiophene groups, the functionalized SiNCs exhibited a redshift of ∼50, ∼65, and ∼115 nm correspondingly (Angi et al., 2018). The in-gap state near the conduction band originated from the aromatic groups was responsible for the redshifts. Besides, in some circumstances the PL of some SiNCs even had no relevance with size. Veinot’s group (Dasog et al., 2013) discovered distinctively different PL phenomena between dodecene terminated SiNCs and NH_4_Br or allylamine functionalized SiNCs. The former followed the rules of quantum confinement, but the latter exhibited size-independent blue PL with a constant peak position of ∼415 nm (Figure 5B) (Dasog and Veinot, 2012). This size-independent PL phenomenon was attributed to the charge transfer from the excited state of SiNCs to nitrogen-related surface states in SiNCs. Then the radiative recombination occurred completely at the nitrogen-related states, which had no relevance with the size of SiNCs (Lannoo et al., 1996; Fuzell et al., 2013; Sinelnikov et al., 2017).

Third, surface modification can enhance the absorption of excitation light and thereby the PL intensity. The indirect bandgap of SiNCs leads to weak absorption of light. To overcome this drawback, light-harvesting antenna was proposed, by imitating chlorophyll which collects sunlight and transfers energy to the reaction center. Similarly, antenna, with excellent light absorption efficiency, first absorbed the incident light and then transferred the energy in the form of electrons to the SiNCs. Finally, the electronic excitation energy of SiNCs transformed into light energy and was emitted in the form of photons. The antenna, as a key functioning component during this absorbing-emitting process, was required to be not only with the higher excited state than that of SiNCs, but also with a suitable distance to the SiNCs acceptor. Because the shorter the length of antenna, the higher the transmission efficiency of the absorbed energy (Mazzaro et al., 2015), pyrene chromophores were the most used light-harvesting antennae. After modifying SiNCs with pyrene chromophores (Figure 5C), the dramatic improvement of absorption at 345 nm was observed. The PL of SiNCs functionalized with pyrene chromophores was as 140% brightness as H-terminated SiNCs with the same size (Mazzaro et al., 2015). Besides, SiNCs functionalized with tetraphenylporphyrin Zn (II) chromophores or pyrene exhibited near-infrared PL and long PL lifetime, which promised the potential application of bioimaging (Locritani et al., 2014; Fermi et al., 2015). Since Korgel’s group (Romano et al., 2016) had summarized the characteristics of light-harvesting antennae system comprehensively, this article would not duplicate the detailed descriptions.

Finally, the surface functionalization is not limited to small molecules discussed above. Actually, SiNCs could be incorporated into polymers to make photoluminescent composites, which might be applicable in more versatile devices. For example, SiNCs were dispersed into off-stoichiometric thiol-ene (OSTE) composition followed by UV irradiation to obtain the SiNCs/OSTE hybrids. The comparatively high QY of ∼65% was observed for SiNCs/OSTE hybrids, which was even higher than the same SiNCs dispersed in toluene solutions. The passivation of SiNCs’ dangling bonds by mobile radicals in the polymer accounted for this excellent optical property (Marinins et al., 2017). In addition, the combination of SiNCs and polymers could also exhibit incredible photostability. The QY of SiNCs/poly(methyl methacrylate) hybrids only reduced from ∼60 to ∼40% after nearly 7 weeks (Marinins et al., 2016). In another research, the polystyrene matrix improved the alkali resistance of SiNCs (Yang et al., 2014). Thanks to the indirect band-gap structure, the SiNCs’ optical transition near the emission state was very weak, which led to the large Stokes shift. Therefore, the composites of SiNCs and polymers generally appeared transparent under the ambient light unlike other semiconductor quantum dots such as CdSe (Figure 5D) (Marinins et al., 2016).

### Temperature During PL Measurement

As described in the previous sections, temperature matters because it is decisive for the size of SiNCs synthesized, but its influence on the PL properties is not confined within the synthetic process. In fact, tuning the temperature during PL measurement serves as a powerful tool for understanding the fundamentals of the PL behaviors of SiNCs. Brus’s group conducted a profound study of the SiNC’s photoluminescence at low temperatures (Wilson et al., 1993). As the temperature decreased from 300 to 20 K, the PL intensity monotonically increased accompanied by a blueshift of peak position. The lifetime of the SiNCs was also increased, but not proportionally to the increment of PL intensity. When the temperature was lower than 50 K, the photoluminescence intensity almost kept constant, but the lifetime was still lengthening. According to Eqs 1, 2 in the previous section, this puzzling phenomenon could be explained. At such low temperature, the radiative recombination term dominated the QY, while the substantially suppressed nonradiative recombination could be ignored. In other words, the emission should purely come from radiative recombination with a theoretical QY of 100%. However, the reality deviated from this hypothesis with the QY of 20%. The possible reason was the existence of defects with extra nonradiative recombination. Besides, the extent of such influence of temperature is contingent on the size distribution. The variation of PL intensity of the smaller SiNCs at low temperature was generally greater than that of the larger ones (Wilson et al., 1993). However, this rule does not apply to SiNCs with a large size in the weakly confined regime (Jakob et al., 2019). For instance, the dramatical drop of PL lifetime was observed starting from above 10–20 K for 4.2 nm SiNCs, but the drop of PL lifetime was not observed until the temperature rose to 150 K for 9.0 nm SiNCs (Takeoka et al., 2000). Meanwhile, at lowered temperature, the PL peaks of SiNCs with a relatively large diameter of 7.19 and 8.67 nm would redshift instead of blueshift (Figure 6) (Jakob et al., 2019). Besides, their mean decay time significantly increased upon cooling. Strangely, the PL intensity of 8.67 nm SiNCs decreased in the range of 700–950 nm, but increased in the range of 950–1,100 nm when the temperature fell. These puzzling phenomena could hardly be explained by a single theory. Perhaps a combination of bandgap widening, saturation effects, and Förster resonance energy transfer (FRET) may help the interpretation (Jakob et al., 2019).

**FIGURE 6:** **(A)** PL peak energy and **(B)** PL peak shift relative to the peak energy at 300 K versus SiNCs’ size at selected temperatures reprinted with permission from Jakob et al. (2019). Copyright 2019 Wiley-VCH Verlag GmbH & Co. KGaA, Weinheim.

## Applications

As discussed in the previous sections, SiNCs obtained by the thermal disproportionation generally exhibit size-dependent PL which is originated from their intrinsic band-gap (Sun et al., 2016a). The most efficient PL emission often falls within the near-infrared which fits the biological windows (Sun et al., 2016b). Moreover, not only the luminescent range but also the PL lifetime of SiNCs is susceptible to the surface species. Therefore, these characteristics have made bioimaging, sensor, and some luminescent devices the most viable applications for SiNCs synthesized from thermal disproportionation.

### Sensor

Exploring new methods to enhance the PL intensity of SiNCs has always been the subject for the researches mentioned previously. However, thinking out of the box, quenching the PL rather than boosting it is not always detrimental, especially in the case of sensors. For instance, the PL of dodecyl functionalized SiNCs was quenched when they were in contact with nitroaromatic compounds such as nitrobenzene, nitrotoluene, and dinitrotoluene (Gonzalez et al., 2014). The quenching process was a dynamic process via electron transfer which occurred from the conduction band of SiNCs to the vacant π* orbital of the nitroaromatic compounds. Based on this mechanism, the dodecyl functionalized SiNCs dispersed in toluene solution can be dip-coated onto the filter paper to fabricate SiNCs sensors for detecting nitroaromatic compounds. When the sensor paper was exposed to nitroaromatic compounds, whether in the form of gas, liquid, or solid, the contact area exhibited significantly suppressed luminescence under the irradiation of UV (365 nm) lamp compared with other luminescent parts. This sensor paper provided an extra choice for on-site detection of explosives that contained nitrogroups. Based on the similar quenching mechanism, SiNCs sensors for other compounds were also investigated. Combining the SiNCs and mAmetrine1.2 (a protein variant), a SiNCs sensor was produced for *p*-nitrophenyl-containing organophosphate nerve agents paraoxon (PX) and parathion (PT). This sensor in the form of paper exhibited high sensibility such that the detection limitation for the concentration was as small as 5 μΜ (Figure 7A) (Robidillo et al., 2019). Besides the sensors for direct detection, some other sensors based on SiNCs synthesized from thermal disproportionation required multiple steps for detection. Veinot’s group demonstrated that the conjugation of urease with SiNCs would first catalytically resolve urea into ammonia, which would quench the PL of SiNCs (Robidillo et al., 2018). In this way, the urea could be detected.

**FIGURE 7:** **(A)** Images of SiNCs coated filter paper spotted with PX and a blank control under the irradiation of UV light (365 nm), reprinted with permission from Robidillo et al. (2019). Copyright 2019 American Chemical Society. **(B)** SiNCs loaded SLN within the MDA435 human breast cancer cells emitted red PL under the irradiation of 458 nm light, reprinted with permission from Henderson et al. (2011). Copyright 2011 WILEY-VCH Verlag GmbH & Co. KGaA, Weinheim. **(C)** Schematic representation of the device containing allylbenzene-capped SiNCs (AB-ncSi) as the emissive layer, reprinted with permission from Mastronardi et al. (2012). Copyright 2012 WILEY-VCH Verlag GmbH & Co. KGaA, Weinheim. **(D)** Illustration of SiNCs-polymer Fabry-Pérot microresonator and **(E)** the spectra of SiQD-polymer hybrid/blend with (solid line) or without (dashed line) Fabry-Pérot cavity structure, reprinted with permission from Cheong et al. (2021). Copyright 2021 American Chemical Society.

### Bioimaging

Integrating the merits of biological compatibility, high PL intensity, and long PL lifetime, SiNCs attracted a lot of attention in the field of bioimaging (Li and Zhu, 2013). In order that SiNCs could be localized in specific tissues or organs, the dispersibility in water and selective absorption by tissue were required. Therefore, it was crucial to functionalize the SiNCs with proper organic groups. For example, SiNCs obtained by the pyrolysis of (HSiO_1.5_)_n_ were first functionalized with 1-octadecene to ensure NIR PL of SiNCs. Then, alkyl-capped SiNCs were covered by the matrix of PEG to form surface-functionalized solid lipid nanoparticles (SLN) in order to realize colloidal stability. As for the cell experiments, clear NIR emission could be observed for human MDA435 breast cancer cells which contained SiNCs (Figure 7B) (Henderson et al., 2011). In addition to the two-step treatment of SiNCs mentioned above, SiNCs could be simply functionalized with specific capping groups that ensure both the colloidal stability and biocompatibility. Veinot’s group demonstrated that the SiNCs terminated with D-mannose and L-alanine, respectively, both exhibited comparable PL for biological imaging of MCF-17 human breast cancer cells (Zhai et al., 2014). The control experiment was performed by exposing cells to pentanoic acid functionalized SiNCs with the aim of investigating if mannose or alanine functionalization could induce cells’ phagocytosis. A positive result that the uptake of mannose and alanine functionalized SiNCs instead of pentanoic acid functionalized SiNCs by the MCF-17 human breast cancer cells was obtained, indicating the multifunctions of D-mannose and L-alanine.

### Other Applications

Apart from the two applications mentioned above, SiNCs are also good candidates for photon manipulations as photosensitizers. This is often realized via the energy transfer from the lowest energy state of the exciton generated in SiNCs to the ground triplet state of oxygen molecules adsorbed on their surface. The long lifetime and huge surface area of SiNCs were beneficial for the high photosensitizing efficiency to generate ^1^O_2_ at room temperature (Llansola Portoles et al., 2010). To further enhance the singlet oxygen generation of SiNCs, the SiNC-dye conjugates were investigated. The SiNCs absorbed near-UV radiation and then transferred this energy to the triplet state of the attached dyes, which increased the number of triplet states and finally enhanced the singlet oxygen generation (Beri et al., 2020). As a reactive oxidant, singlet oxygen exhibited great potential for quantities of applications, such as chemical synthesis (Manfrin et al., 2019; Karsili and Marchetti, 2020), environmental protection (García-Fresnadillo, 2018; Bu et al., 2021), and photodynamic therapy (Guo et al., 2010; Bartusik-Aebisher et al., 2021; Osuchowski et al., 2021), and thus the application fields of SiNCs were also broadened.

Photonic devices have always been another sought-after field for SiNCs with high QY value and solution processibility after functionalization. In order to reduce the environment toxicity of LED industry, SiNCs were considered as replacement for CdSe and PbS (Puzzo et al., 2011), and the surface modification with organic groups such as allylbenzene could effectively improve their poor EQE as OLEDs (Figure 7C) (Mastronardi et al., 2012a). Besides, carrier multiplication was observed in silicon, which would dramatically enhance the photovoltaic efficiencies for solar cells (Timmerman et al., 2011). Sukhanov’s group indicated that the 12% increase of power conversion efficiency of silicon quantum dot solar cell came from the defect passivation at the surface of solar cell by SiNCs and the decrease of the optical reflectance (Dorofeev et al., 2014; Gribov et al., 2018). Engineering the bandgap of SiNCs can further improve the solar cell efficiency. A novel stepwise bandgap SiNCs layer structure was put forward, which was composed of a top layer (high bandgap) and a bottom layer (low bandgap). This combination improved charge transfer efficiency, and hence the power conversion efficiency of SiNCs solar cell was also increased from 16.50 to 17.50% compared to the efficiency of solar cell with uniform bandgap structure (Kwak et al., 2017; Kwak et al., 2020). In addition to the PL intensity, PL line width also played a critical role in light-emitting devices. A novel structure with Fabry−Pérot resonators was put forward (Cheong et al., 2021). By incorporating SiNCs-polymer hybrid/blend between two reflective silver mirrors (Figure 7D), the devices obtained an incredibly narrow spectral bandwidth of 9 nm, which revealed its potential for color filter application (Figure 7E). Without modification process, the H-terminated SiNCs could be used for luminescence patterning or optical storage because of the photoactivation by blue or UV irradiation. Exposing the H-terminated SiNCs under UV irradiation for a few minutes, their PL intensity would increase dozens of times (Lockwood et al., 2011). Other applications such as lasers were also investigated by researchers because of the distinctive optical gain of SiNCs embedded in SiO_2_ with a broad gain curve ranging from 650 to 850 nm (Pavesi, 2000; Liang and Bowers, 2010; Koshel et al., 2011). Again we would like to state that the applications of SiNCs would never be limited within the cases discussed above, and here we only highlight some of those employed SiNCs synthesized from the thermal disproportionation reaction.

## Conclusion and Outlook

With the continuous development of SiNCs’ research, the relationship between structure and PL properties of SiNCs has been gradually revealed, which has spawned the design of novel SiNCs-based materials with excellent PL performance and in turn the potential for wide application and industrial production. For the synthesis of SiNCs, thermal disproportionation offers an excellent choice, by integrating the merits of feasible production, precise controllability of size, PL emission from the bandgap, and availability for further surface modification. There is a toolbox of approaches to tune the PL of SiNCs synthesized with this method. The most straightforward ways are to adjust the size of SiNCs under the guidance of quantum confinement effects, such as tuning the heating temperature, heating time, Si/O ratio, and the structure of precursors. Apart from the size of SiNCs, defects generated at the interface of SiNCs and concomitant SiO_2_ also play an important role to abate PL as nonradiative recombination centers. In this regard, hydrogen and oxygen passivation are effective methods to eliminate defects, and some organic capping groups exhibit similar functions. Besides, a wide variety of capping groups enrich the possibilities of SiNCs. Through surface reactions like hydrosilylation, functionalized SiNC are endowed with biocompatibility and tunability in both emission wavelength and intensity, meeting different targeted application requirements.

However, thermal disproportionation is not flawless. First of all, the Si/O ratio of the raw materials limited the production yields of SiNCs. For SiO, the maximum atomic conversion of Si is 50% theoretically, and the actual yield would be much lower than 50%, considering that the majority of the product is still the matrix of SiO and SiO_2_ which gains all the weight of O and half of the Si, and the conversion would never be complete. Next, to release the SiNCs from the matrix, HF etching is usually required, which might be a cumber and hazard to nonchemists. Finally, high heating temperature during the thermal disproportionation requires extensive energy consumption, resulting in high cost and significant carbon footprint.

While not being impeccable, thermal disproportionation is a prevailing and solid technique to yield luminescent SiNCs, towards which the understanding may lead to the design and implementation of more viable photonic and biocompatible applications. We envision several potential directions for its further developments. First, more versatile compositions of the silicon-rich oxides through introduction of metal elements and inorganic components could endow SiNCs with new catalytic behaviors (Wong et al., 2017; Sun et al., 2020). For example, Ti-doped silicon nanocages would enhance their catalytic performance for CO_2_ hydrogenation because of the unsaturated electronic states of silicon cage, which was originated from the strong covalent bonding between Si and Ti (Pei et al., 2019; Wu et al., 2020).

Second, hybridizing the precursor with suitable solvents and polymers could offer compatibility with conventional printing and the novel 3D printing techniques, which in turn renders patterning of the luminescent Si structures possible. As a recent example demonstration, hybrid dots of silicon and carbon combined with binders were invented as anticounterfeiting inks, which could be applied to various substrates for printing, including yarns, cotton fabric, cellulosic paper, glass, metal, silicon wafer, and PET film (Fu et al., 2021; Lyu et al., 2021). The highly saturated color of the inks could also be realized by Mie resonance of silicon nanoparticles (Sugimoto et al., 2020; Okazaki et al., 2021). Besides, the combination of 3D printing technique and quantum dots could enable the fabrication of optoelectronic devices with complex structures (Chen et al., 2020a; Xu et al., 2021b). By incorporating the silicon quantum dots into the 3D printed devices, the hybrids could be more biocompatible and environmentally benign.

Third, photosensitizers for upconversion have drawn increasing attention recently. Similar to the photosensitizers mentioned in *Other Applications* section for singlet oxygen generation, silicon quantum dots absorb light energy and convert it to the spin-triplet excitons centered on molecules bound to their surface. By functionalizing SiNCs with 9,10-diphenylanthracene ligands, the SiNCs obtained could upconvert 488–640 nm light to 425 nm violet light (Xia et al., 2020). However, the quenching of triplet excitons by oxygen hindered further development of SiNCs with the property of light upconversion. To strengthen the stability, polymer barriers on SiNCs’ surfaces to retard the diffusion of oxygen has been demonstrated as a viable solution (Xia et al., 2021). Moreover, bidirectional triplet exciton transfer could also be realized by functionalizing SiNCs with perylene chromophores (Huang et al., 2021). Despite the fact that the SiNCs employed in these works were synthesized via nonthermal plasma, we are confident that SiNCs generated from thermal disproportionation should exhibit similar behaviors.

Fourth, electronic devices have been an unfading field of SiNCs (Ni et al., 2019). Besides the traditional SiNCs light-emitting devices and photovoltaics, the new-generation optoelectronic synaptic devices have been demonstrated. For example, synaptic transistors structures that combined the perovskite and SiNCs exhibited the increased optical sensitivity and decreased electrical energy consumption (Yin et al., 2020; Zhu et al., 2020). We expect that SiNCs could find their use in more novel forms of devices, e.g., related to data storage, laser, and amplifiers (Dohnalova et al., 2014).

Finally, classical silane and organosilicon chemistry is still a treasure house to refer to (Dasog et al., 2016; de Almeida et al., 2021), for the endless ways of surface modifications of SiNCs freed from the oxide matrix, which could confer a myriad of new functionalities on them, enabling unforeseen but exciting applications.
